The article "Exploring Effects of Sensory Garments on Participation of Children on the Autism Spectrum: A Pretest-Posttest Repeated Measure Design" was published in 2022. Journal: Occup Ther Int.

# Exploring Effects of Sensory Garments on Participation of Children on the Autism Spectrum: A Pretest-Posttest Repeated Measure Design

**DOI:** 10.1155/2022/3540271

**Published:** 2022-06-06

**Authors:** Lisa Mische Lawson, Lauren Foster, Kayla Hamner, Lacy Wright

**Affiliations:** Department of Occupational Therapy Education, University of Kansas Medical Center, USA

## Abstract

**Objective:**

Autistic children experience sensory challenges that interfere with participation and increase parent stress. Sensory-based interventions are used to address children's behaviors affected by sensory processing difficulties, but research is limited regarding use of sensory garments to support participation of autistic children. This study explored sensory garment effects on participation, parental competence, and perceived stress of autistic children and their parents.

**Method:**

Twenty-one children were recruited and 17 males with ASD and atypical sensory processing patterns completed the 14-week study. The Canadian Occupational Performance (COPM) and Goal Attainment Scaling (GAS) were used to set and monitor participation goals. After a baseline period, children wore sensory garment(s) for 8 weeks. The COPM, GAS, Parent Stress Index-Short Form (PSI-SF), and Parent Sense of Competence Scale (PSOC) were administered four times (prebaseline, before and after the intervention, and three weeks postintervention).

**Results:**

There were moderate to large significant differences in both COPM and GAS scores after the intervention and from the beginning to the end of the study indicating sensory garments may improve participation of autistic children. There were no significant differences in PSI or PSOC at any timepoint. Two children rejected the garments.

**Conclusions:**

Parent- or child-selected sensory garments may improve participation in individually meaningful activities for children who can tolerate wearing them. Children's improvement in participation did not improve parent stress or competence, possibly due to the passive nature of the intervention. More research is needed explore the influence of heterogeneous sensory patterns on response to intervention.

## 1. Introduction

Autism Spectrum Disorder (ASD) is a developmental disorder that impacts 1 in 44 children nationally [1]. Many autistic children exhibit different sensory processing patterns compared to typically developing peers [2]. Sensory processing refers to the ability to interpret and respond to sensory input [3, 4], and participation problems may arise when a mismatch exists between a person's environment and their sensory processing pattern. Sensory processing differences in autistic children may include increased sensitivity (hyperresponsivity) or decreased sensitivity (hyporesponsivity) to various environmental stimuli [5]. Evidence suggests that these differences can impact children's participation across various contexts and influence the daily activities in which families choose to engage [6, 7]. For example, autistic children may engage in repetitive or stereotyped movements, such as rocking, spinning, and fidgeting, or may cover their ears, not respond to their name, or even elope [8]. These behaviors are associated with efforts to regulate the sensory system by avoiding or seeking sensory input [9] and may limit participation in play, school, social activities, and self-care [6, 10].

The article "Exploring Effects of Sensory Garments on Participation of Children on the Autism Spectrum: A Pretest-Posttest Repeated Measure Design" was published in 2022. Journal: Occup Ther Int.

Evidence shows parents of autistic children experience more stress than parents of typically developing children or children with another disability [11, 12]. This increased parenting stress may be associated with the daily responsibilities of caring for an autistic child who exhibits challenging behaviors [11]. Such behaviors may contribute to parent stress due to cultural expectations for parents to manage their child's inappropriate or disruptive behaviors [12]. In addition to stress, family activities and routines across different contexts are largely influenced by children's everyday participation [7, 10]. Due to their child's sensory processing difficulties, families tend to adhere to organized routines, avoid overstimulating or understimulating environments, and prepare backup plans to prevent behavioral disruptions, especially during community activities [10, 13]. Particularly, hyperresponsiveness to sensory stimuli has been found to have a negative effect on participation in social and community occupations, likely due to these settings being unpredictable and not easily controllable by parents [10]. Therefore, utilizing interventions that address sensory processing may improve participation for children in addition to supporting parent outcomes.

Sensory-based interventions are often used to address children's behaviors affected by sensory processing difficulties [13, 14]. Sensory-based interventions may incorporate weighted vests, weighted blankets, sensory diets, and sensory garments to support sensory processing differences. Theoretically, when integrated into daily routines, these methods may improve self-regulation, promote activity, and reduce over reactivity [13]. While these supports may be beneficial for children, recent literature suggests that weighted vests and weighted blankets do not have a significant impact on outcomes such as repetitive behaviors, joint attention, and distractibility in autistic children [13, 15, 16]. A lack of consistent evidence on the overall effects of sensory supports for autistic children calls for further investigation into sensory-based interventions, specifically related to activity participation in children and their families. Furthermore, the sensory processing profiles of autistic children vary [17], yet research of sensory-based interventions often does not consider the heterogeneity of sensory processing of autistic children when investigating response to intervention [18].

The article "Exploring Effects of Sensory Garments on Participation of Children on the Autism Spectrum: A Pretest-Posttest Repeated Measure Design" was published in 2022. Journal: Occup Ther Int.

Literature shows mixed results for sensory interventions, and research on various sensory garments as a primary support for sensory processing is limited. Compression garments are one type of deep pressure intervention that may help regulate the sensory system through pressure applied to the body [19, 20]. As these garments distribute pressure evenly on the body compared to weighted vests which localize pressure to the shoulders, they may promote increased body awareness and focus. Compression garments can be incorporated into daily routines and support both child and parent preferences [21]. Other types of sensory garments, including seamless options, may also improve children and family outcomes, though evidence on their use is minimally available. Kabel et al. [22] suggest autistic children who demonstrate stress from sensory-agitators (i.e., sensory stimuli they find aversive) may benefit from sensory-sensitive clothing that consider seams and materials [22]. The researchers also state that parents of autistic children expressed concerns with the current accessibility of sensory-sensitive clothing options. Therefore, for this study we examined the effectiveness of sensory garments in (1) increasing occupational participation of autistic children and (2) increasing parental competence and reducing perceived stress.

## 2. Method

### 2.1. Research Design

We used a pretest, posttest repeated measures design for 14 weeks to examine if SmartKnitKIDS sensitivity garments resulted in increased child participation and parental competence, while decreasing parent stress. This study was approved by University of Kansas Medical Center institutional review board (#00146392) and carried out in accordance with the Declaration of Helsinki as revised in 2000. Parents provided informed consent, and children assented to participation when parents determined they were capable. Participants received incentive for completing all study activities.

### 2.2. Participants

We aimed to recruit a convenience sample of twenty children due to practical constraints of the study. Participants were recruited through departmental research lists, social media (e.g., closed Facebook Autism groups), child development centers, private practice, and word of mouth over four months. Children were included if they were ages 4-17, had a Social Responsiveness Scale score greater than 62, if the Child Sensory Profile-2 indicated at least one sensory pattern outside “typical” (e.g., more or much more or less than others), and parents indicated unmet needs within family life. Children were excluded from the study if they did not meet the inclusion criteria.

The article "Exploring Effects of Sensory Garments on Participation of Children on the Autism Spectrum: A Pretest-Posttest Repeated Measure Design" was published in 2022. Journal: Occup Ther Int.

### 2.3. Measures

This study used screening measures to determine eligibility and an assessment battery to determine intervention effectiveness. Participants completed the measures from their home via Zoom or REDCap.

#### 2.3.1. Screening Measures

*(1) Social Responsiveness Scale-2 (SRS-2)*. The SRS-2 is a 64-item caregiver report of autism severity [23]. It has good internal consistency (.94-.96) and test-retest reliability (.88-.95) and has been found to have strong concurrent validity with the Child Autism Rating Scale [24]. A cut-off score of 62 identifies 96.8% of autistic children and yields sensitivity and specificity values of .92. The SRS-2 was used to confirm parent-reported autism diagnosis.

*(2) Child Sensory Profile-2 (CSP2)*. The CSP2 is a caregiver reported questionnaire with 86 questions related to sensory preferences in children ages 3-14 years [3]. The assessment provides scores for four sensory processing quadrants (registration, seeking, sensitivity, and avoiding), six sensory sections (auditory, visual, touch, movement, body position, and oral), and three behavioral sections (conduct, social-emotional, and attentional). The CSP2 demonstrates good validity (*α* = .60 − .90), reliability (.87-.97), and goodness of fit (*χ*^2^ = 15,412.588, *p* < .000) for the four sensory processing quadrants [25].

#### 2.3.2. Assessment Battery

*(1) Canadian Occupational Performance Measure (COPM)*. The COPM is an assessment in which caregivers identify concerns related to self-care, productivity, and leisure [26]. Parents rated children's levels of performance and satisfaction on a scale of 1-10. The COPM has adequate internal consistency for performance (.56) and satisfaction (.71) scales and good test-retest reliability (.80) [27]. Based on the top five identified concerns, parents developed a participation-related goal with an interventionist.

*(2) Goal Attainment Scaling (GAS)*. GAS measures progress toward individualized, meaningful goals and is a helpful outcome measure in autism studies with broad eligibility criteria [28]. GAS uses a scale of -2 to +2, with 0 assigned as baseline for this study, -2 reflects goal behaviors worsening, and +2 represents goal behaviors improving. A review of 52 pediatric studies showed GAS to be a clinically useful tool for measuring progress toward goals [29].

*(3) Parent Stress Index-Short Form (PSI-SF)*. The PSI-SF is a 36-item questionnaire for parents to indicate responses to life events using a 5-point Likert Scale (1 = strongly disagree to 5 = strongly agree), with higher scores indicating greater stress [30]. Cronbach's *α* of subscales range from.80 to .88 indicating adequate reliability, and the parent distress subscale is considered useful for measuring distress in parents of autistic children [31].

*(4) Parent Sense of Competence Scale (PSOC)*. The PSOC is a 17-item scale (1 = strongly disagree to 6 = strongly agree) that measures parental self-efficacy and satisfaction, with higher scores indicating greater sense of competence [32]. Internal consistency of the scale with autism populations is high (Cronbach's *α* .74-.76), and it has been widely used in studies to evaluate parenting self-esteem, efficacy, and competence [33].

The article "Exploring Effects of Sensory Garments on Participation of Children on the Autism Spectrum: A Pretest-Posttest Repeated Measure Design" was published in 2022. Journal: Occup Ther Int.

### 2.4. Intervention

Two occupational therapists and five occupational therapy graduate students provided the testing and intervention for the study. The interventionists met with participants virtually using a HIPPA complaint platform. All sessions were video recorded. Intervention meetings and communication with families were documented and saved for intervention fidelity.

Table 1 illustrates the timeline for intervention and data collection. For test 1, researchers met with families to complete the COPM and GAS to determine familial daily routines and collaboratively set goals. Then, a 3-week waiting period took place where no interventions were provided other than those already in place. During test 2, researchers and parents reviewed GAS and reassessed important occupations identified through the COPM in addition to choosing a sensory garment to wear that would support their goal. Parents and children could choose to wear one or more of the following SmartKnitKIDS seamless products: (1) sensitivity socks, (2) Compresso-T, (3) bralette, (4) undies, and/or (5) compression sleeve [34]. In the 8-week intervention period, participants wore the chosen sensory garments and researchers conducted weekly check-ins with parents. Throughout these weekly check-ins, researchers monitored progress, adjusted goals or garments if needed, and provided support for wearing the sensory garments. Interventionists only provided guidance on garment wearing and provided no other sensory-based intervention recommendations. At the end of the 8 weeks, researchers and families completed the assessment battery for test 3. Test 4 assessment battery occurred 3 weeks later. The time between test 3 and test 4 was a 3-week waiting period in which participants were given the option to continue wearing the garments. At each test phase, parents completed the PSI-SF and PSOC to assess responses to life events, parental self-efficacy, and satisfaction. The study ended when all participants had completed the follow-up measures.

The article "Exploring Effects of Sensory Garments on Participation of Children on the Autism Spectrum: A Pretest-Posttest Repeated Measure Design" was published in 2022. Journal: Occup Ther Int.

#### 2.4.1. Intervention Fidelity

The licensed therapists trained and provided supervision to the five graduate students. The primary investigator (PI) was not an occupational therapist, did not participate in the assessment or intervention process but provided general oversight. The PI also provided written and online training for the research protocol, including the intervention. The research team met weekly to debrief and ensure they were administering assessments and providing the intervention consistently. During these meetings, researchers documented their decision-making process related to the research procedures.

### 2.5. Data Analysis

We used descriptive statistics to summarize demographic characteristics of our sample. We used a within-subject repeated measure analysis of variance (ANOVA) or Friedman's ANOVA (nonparametric data) to determine effects for time [35]. We made four comparisons:

1. TIME 1–TIME 2 (baseline): Do outcomes change over a 3 wk wait period with no intervention?
2. TIME 2–TIME 3: Is the intervention effective?
3. TIME 3–TIME 4: Are effects sustained?
4. TIME 1–TIME 4: Are there overall changes from first to last meeting?

We used Bonferroni correction to control for familywise error, adjusting our significance level to *p* < .0125. We used planned contrasts and Wilcoxon post hoc testing (nonparametric data) to identify where differences were significant when there was an overall significant effect. We used Eta squared, Hedge's *g*, and Kendall's *W* to report effect size. Hedge's *g* is like Cohen's *d* but better corrects for upward bias with sample sizes below 20 [36].

## 3. Results

### 3.1. Sample Characteristics

Twenty-one families were recruited to the study. One child did not have an atypical sensory pattern and was excluded, one parent dropped out after the baseline period without providing a reason, and two children (one male, one female) refused to wear the garments, specifically the tank top and were excluded from analysis. Those refusing the Compresso-Ts, described them as “itchy,” “too tight,” and “too difficult to put on.” The final sample included 16 parents and 17 children as one sibling pair participated in the study.

All the child participants were male, and most were Caucasian (*n* = 9) with average age 7.9 years (SD = 3, range 4-13). SRS scores indicated that most children (*n* = 12) had severe social impairments, six took medication, and all children received services with the most common being OT (*n* = 11) and Applied Behavior Analysis (ABA, *n* = 11). Other services included speech (*n* = 8), special education (*n* = 6), psychiatric care (*n* = 4), physical therapy (*n* = 2), and other complementary therapies such as play therapy or hippotherapy (*n* = 3). Children's sensory patterns showed that most had more or much more characteristics across all four sensory quadrants (avoiding, seeking, sensitivity, and registration), and thirteen children had previously tried sensory wearables (see Table 2).

The article "Exploring Effects of Sensory Garments on Participation of Children on the Autism Spectrum: A Pretest-Posttest Repeated Measure Design" was published in 2022. Journal: Occup Ther Int.

### 3.2. Goal Attainment Scale

Goals for the 17 children were related to sleep (*n* = 7), dressing (*n* = 5), both sleep and dressing (*n* = 1), play (*n* = 2), academics (*n* = 1), and community safety (*n* = 1). Sleep goals included settling down, falling asleep, and staying in bed. Dressing goals included selecting clothes, dressing more quickly, and keeping on clothing. The Friedman test revealed a moderate, significant difference between GAS scores by time (*X*^2^(3) = 21.508, *p* < .001, *W* = .422). Wilcoxon post hoc tests showed significant differences with small-moderate effect from time2-time 3 (intervention, *p* = .010, *W* = .318) and large effect from time 1-time 4 (overall effects, *p* = .007, *W* = .605). There were no significant differences between any other testing times.

### 3.3. Canadian Occupational Performance Measure

There were large, significant differences by time in COPM performance (*F* = 8.424, *p* = .000, *ƞ*^2^ = .283) and satisfaction scores (*F* = 11.786, *p* = .000, *ƞ*^2^ = .356). Like the GAS, post hoc tests showed large, significant differences from time 2-time 3 (intervention) and time 1-time 4 (overall effects). There were no significant differences between any other testing times.  Table 3 shows significance and effect size of all COPM performance and satisfaction planned comparisons.

### 3.4. Parent Stress and Sense of Competence

There were no overall significant differences by time for PSI and PSOC total scores (*F* = .581, *p* = .630; *F* = .391, *p* = .760) and subscale scores (PSI defensive responding, *F* = 1.010, *p* = .394; PSI parental distress, *F* = 1.027, *p* = .387; PSI dysfunctional interaction, *F* = .233, *p* = .873; PSI difficult child, *F* = .298, *p* = .827; PSOC satisfaction, *F* = .416, *p* = .742; PSOC efficacy, *F* = .840, *p* = .477; and PSOC interest, *F* = .813, *p* = .492), so post hoc planned comparisons were not conducted.

## 4. Discussion

This study explored the effects of sensory garments on occupational participation of autistic children. Findings suggest that parent- or child-selected sensory garments may improve participation in individually meaningful activities, particularly sleep and dressing, for children who can tolerate wearing them. This is consistent with evidence showing interventions focused on supporting families to achieve their prioritized goals lead to significant and meaningful improvement in children's participation [37]. However, our positive findings are inconsistent with previous research investigating sensory wearables (e.g., weighted vests) for which evidence supporting their use is limited [15] and reports few positive effects [13]. Some parents in this study set goals with their child, and collaborative goal setting is known to increase self-determination of children with disabilities leading to better goal attainment [38]. Additionally, goal setting is known to direct attention toward the goal and energize behavior change [39], so it is possible that parents and children in the current study benefitted from the process of setting and evaluating progress toward participations goals rather than children benefitting from the sensory garments. Conversely, the significant, meaningful changes in participation goals occurred only during the intervention period and from the beginning to end of the study which may suggest that the garments had some effect.

The article "Exploring Effects of Sensory Garments on Participation of Children on the Autism Spectrum: A Pretest-Posttest Repeated Measure Design" was published in 2022. Journal: Occup Ther Int.

Previous research suggests that parent stress decreases and Parent Sense of Competence increases when children make progress toward individualized, meaningful goals [37]. Though children made progress toward goals in the current study, there was no improvement in parent stress and sense of competence. This may be due to the relatively passive nature of our intervention (e.g., selecting and encouraging wear of a sensory garment). It is possible that parents need to be actively engaged in the intervention process to increase competence and decrease stress, such as the coaching process in the Dunn et al. study (2012) that encouraged parents to come up with their own solutions. Additionally, the use of sensory garments as an intervention did not include an educational component that previous research has shown to be helpful for improving parent stress [40] nor did it consider the environmental or behavioral aspects necessary for improving parent stress [41]. Since autistic children thrive on routine, parent stress may have been impacted by change in routine to introduce the sensory garments [10, 13] or the potential burden of research participation [42]. Current study findings challenge the assumption that child progress will positively impact parent outcomes.

It is important to note that one participant discontinued the study for unknown reason prior to introduction of the sensory garments, and two children would not wear the sensory garments. It is possible that ill-fitting or nonpreferred sensory garments could exacerbate negative behaviors and worsen participation. Research indicates autistic children tend to be sensitive to the type of clothing worn [43]. In the current study, children's sensory preferences may not have been compatible with the garment, or they may have been better supported by change of size or fabric. Previous research has not investigated the heterogeneity of sensory preferences related to effectiveness of sensory interventions [17], so it is also possible that specific sensory preferences are not a good match for use of sensory garments, particularly compression garments like the ones children rejected in this study.

The article "Exploring Effects of Sensory Garments on Participation of Children on the Autism Spectrum: A Pretest-Posttest Repeated Measure Design" was published in 2022. Journal: Occup Ther Int.

### 4.1. Future Research

Future research should seek to better understand how sensory preferences influence response or nonresponse to sensory interventions. A larger sample adequately powered to explore the effects of sensory differences on results would be beneficial. Researchers might also consider qualitative or mixed-method research to investigate the perspectives of children who reject or cannot tolerate sensory garments. Future research should also include a comparison group to control for potential bias related to expectation effect.

### 4.2. Implications for Practice

Due to the exploratory nature of the study, the results should be considered with caution. However, these results have several possible implications for occupational therapy practice. First, this study illustrates the importance of collaborative goal setting between the parent and therapist. Second, understanding children's unique sensory preferences through consultation with an occupational therapist could be helpful for selecting and introducing sensory garments. Third, parents and professionals should consider children's and families' tolerance for change before introducing sensory garments. Fourth, several options and sizes should be provided to ensure that the garments are preferred and offer comfortable fit. Finally, because we know little about why children refuse or cannot tolerate sensory garments, parents and therapists might carefully consider if and how long they want to try them with autistic children.

### 4.3. Strengths/Limitations

A strength of our study was investigating the use of commercially available sensory garments in the natural environment as parents would be most likely to use them with their children. Additionally, our sample was heterogeneous in terms of age, ethnicity, medication use, sensory preference, and severity of autism. However, our sample was limited to only males, and we did not have adequate sample size to explore if differences in how sensory preferences influenced the results. Additionally, our volunteer sample of parents may have been more motivated to follow through with goals than the general population of parents of autistic children. Because blinding was not possible, expectation bias may have occurred. Participants reported high COPM ratings for both satisfaction and performance at time 3 after the intervention, leaving little room for improvement at time 4 indicating possible ceiling effect. Even with these limitations, this study advances the limited knowledge related to sensory wearables that are popular in the autistic population.

The article "Exploring Effects of Sensory Garments on Participation of Children on the Autism Spectrum: A Pretest-Posttest Repeated Measure Design" was published in 2022. Journal: Occup Ther Int.

## 5. Conclusion

Autistic children experience sensory challenges that interfere with participation and increase parent stress. Though there is limited evidence regarding their effectiveness, sensory-based interventions (i.e., sensory garments) are often used to address children's behaviors affected by sensory processing difficulties. This pre-post repeated measures design study contributes to the body of evidence regarding the use of sensory garments with autistic children. This study found that parent- or child-selected sensory garments may improve participation in individually meaningful activities for children who can tolerate wearing them. Additional studies are needed to explore child characteristics related to best response. Occupational therapy sensory assessment and consultation could be valuable for caregivers considering sensory garments for autistic children.

### 5.1. Language Usage

The authors recognize that the use of identity-first language is not universally accepted and may not reflect the beliefs of individuals who participated in our study. We chose to use identity-first language based on recent research in the United States and the United Kingdom showing that this language is preferred by the majority of autistic individuals and their families who responded to the surveys.

## Figures and Tables

**Table 1:** Timeline of intervention and data collection.

Time 1	Waiting period 3 weeks	Time 2	Intervention period 8 weeks	Time 3	Waiting period 3 weeks	Time 4
COPM GAS PSI-SF PSOC	Baseline	COPM GAS PSI PSOC	Wear garment Weekly check-in documentation	COPM GAS PSI-SF PSOC	Sustainability	COPM GAS PSI-SF PSOC

*Note*. COPM: Canadian Occupational Performance Measure; GAS: Goal Attainment Scale; PSI-SF: Parent Stress Index-Short Form; PSOC: Parent Sense of Competence.

**Table 2:** Participant demographics.

Participant characteristics	Number (%)
Age	
4-6 years	6 (35.3)
7-9 years	7 (41.2)
10-13 years	4 (23.5)
Ethnicity	
Asian	1 (5.9)
Black or African American	2 (11.8)
Caucasian	9 (52.9)
Hispanic or Latino	1 (5.9)
Multiple ethnicities	4 (23.5)
Diagnosis	
Autism	11 (64.7)
Asperger syndrome	1 (5.9)
Dual diagnosis^∗^	5 (24.9)
Social Responsiveness Scale category	
Mild	1 (5.9)
Moderate	4 (23.5)
Severe	12 (67.0)
Previous sensory wearables	
None	4 (23.5)
Weighted vest	3 (17.6)
Weighted blanket	3 (17.6)
SPIO smart knit shirt	2 (11.8)
Soft stretchy materials	1(5.9)
Multiple sensory garments/items	4 (23.5)
Sensory preferences	
Avoiding	
Like others	6 (35.3)
More than others	6 (35.3)
Much more than others	5 (24.9)
Seeking	
Like others	4 (23.5)
More than others	8 (47.1)
Much more than others	5 (29.4)
Sensitivity	
Like others	5 (29.4)
More than others	6 (35.3)
Much more than others	6 (35.3)
Registration	
Like others	4 (23.5)
More than others	2 (11.8)
Much more than others	11 (64.7)

^∗^ *Note.* Diagnoses cooccurring with autism included sensory processing disorder, Down syndrome, global developmental delay, or PACS1 gene mutation.

The article "Exploring Effects of Sensory Garments on Participation of Children on the Autism Spectrum: A Pretest-Posttest Repeated Measure Design" was published in 2022. Journal: Occup Ther Int.

**Table 3:** COPM performance and satisfaction score differences by time.

Within subject effects	df	*t*	*p*	*g*
Time 1–time 2	64			
Performance		-.718	.475	-.243
Satisfaction		-.757	.452	-.257
Time 2–time 3	64			
Performance		-2.465	.016	**-.836**
Satisfaction		-3.161	**.002**∗	**-1.071**
Time 3–time 4	64			
Performance		-1.185	.240	-.402
Satisfaction		-1.113	.329	-.377
Time 1–time 4	64			
Performance		-4.368	**.000**∗	**-1.481**
Satisfaction		-5.030	**.000**∗	**-1.705**

*Note*. ^∗^significant effect; 0.2 = small effect, 0.5 = medium effect, and 0.8 = large effect; significant and large effects bolded.

## Data Availability

Contact the corresponding author for data.
